# Study on Maximal Oxygen Uptake of Respiration and Heart Rate in Exercise Training Based on Regression Equation

This article has been retracted.

**DOI:** 10.1155/2022/5961197

**Published:** 2022-03-10

**Authors:** Yongqing Liang, Qiufen Yu

**Affiliations:** Physical Education College, Qiqihar University, Qiqihar, Heilongjiang 161006, China

## Abstract

To investigate the important index of maximum oxygen uptake in evaluating cardiopulmonary function and to provide a basis for the evaluation of cardiopulmonary function for adolescents, a total of 200 healthy adolescents aged 12–14 were selected, and these 200 subjects were randomly assigned to the modeling group and the test group. In the first stage, data of 150 subjects were randomly selected, and the regression equation for VO2max was established by adding independent variables such as gender, age, height, weight, body mass index, and resting heart rate. In the second stage, the remaining 50 subjects were selected as the test group to test and evaluate the prediction effect of the prediction model. The results showed that the correlation coefficient between the measured value of maximal oxygen uptake and the predicted value was 0.983, and the significance level was 0.000, which was significantly lower than 0.01 correlation, indicating that there was an obvious concomitant relationship between the two values. The maximum oxygen uptake calculated by this equation is good and has a good application prospect.

## 1. Introduction

With the improvement of social living standards, most social groups spend their time on making money and lack physical exercise, especially teenagers who lack exercise or spend enough time on exercise, resulting in unhealthy health [1]. For teenagers, no matter in physical or psychological health, we should pay special attention to their physical health which is closely related to the development of society. Nowadays, there are a large number of factors that affect their physical conditions, and there is an unbalanced development among these factors [2]. The main performance is in the following points: the overall level of teenagers has been greatly improved, but their physical quality is constantly declining. And these physical impairments are now seriously affecting their health. In relevant studies, the physical fitness of primary and secondary school students in China has been comprehensively tested, and continuous research has been carried out on each stage of establishing the index system [3].

There are many studies on predicting the regression equation of maximal oxygen uptake. As there are many influencing factors and related indicators of maximal oxygen uptake, the regression equation of maximal oxygen uptake is different for different groups [4]. By measuring some relevant indexes of subjects through simple tests, the regression equation model that can directly calculate maximal oxygen uptake can be deduced, which is simple and easy to use [5]. Chidnok studied the effect of high circulatory quality on vascular function and cardiopulmonary function in sedentary humans. Methods: twenty-two female participants were divided into two groups, an intervention that did not receive an intervention and a control HIIT group. The medical history of each participant interviewed was collected and recorded, and medical parameters including cardio-ankle vascular index (CAVI), flow-mediated dilation (FMD), and maximum oxygen consumption (VO2MAX) were used as baseline predictors. The intervention was a cyclic HIIT lasting 6 weeks with three sessions per week. During each session, participants completed a 1-minute set protocol on a circulatory dynamometer, cycling at 80–85% of their maximum heart rate, and then rested. The sequence was repeated a total of five times. Results: after 6 weeks of intervention, the results showed that CAVI (6.39 ± 0.76 vs. 5.91 ± 0.58), FMD (9.26 ± 6.5 vs. 14.01 ± 4.3%), and VO2max (20.10 ± 4.31 vs. 24.34 ± 5.71 mL/kg/min) were compared with the predictive test (*P* < 0.05). In addition, HIIT, as measured by FMD, increased endothelial function (14.01 ± 4.3 vs. 9.15 ± 4.16%, *P* < 0.05). Conclusions: six weeks of HIIT was found to improve vascular function and cardiopulmonary function in the poor and demonstrate the benefits of HIIT as a stable exercise strategy [6].

In conclusion, this paper proposes a study on maximal oxygen uptake of respiration and heart rate during exercise training based on regression equation. Choose vo_2_ Max as the dependent variable, gender, age, height, weight, body mass index (bmi), exhausted heart rate, maximum heart rate, load as the independent variable, stepwise regression analysis, the results in these indicators, sex, weight, body mass index, and maximum heart rate, load five indicators into the regression equation, and thus infer teenagers' VO2 Max regression model. The maximum oxygen uptake calculated by this equation is good and has a good application prospect.

## 2. Research Methods

### 2.1. Research Objects

A total of 200 healthy adolescents aged 12–14 were randomly selected for this study. These 200 subjects were randomly assigned to either the modeling group or the test group. Among them, modeling group has150 people and inspection group has50 persons. All subjects completed all tests. Prior to the experiment, informed consent should be signed with the consent of the subjects and their parents. All the students participating in the experimental study have no physical defects, can carry out normal physical exercise, and did not participate in any form of professional sports training. There were no statistically significant differences in age, height, weight, BM work, resting heart rate, exhausted heart rate, maximum heart rate, and maximum load and maximum oxygen uptake between the two groups (gender was represented by code: male = 0 and female = 1).

### 2.2. Methods

#### 2.2.1. Experimental Design

A sports and health questionnaire suitable for adolescents was issued and the subjects of this study were recruited. The par-Q was used to understand the previous medical history and physical activity level of the subjects, and 200 adolescents aged 12–14 were selected as subjects of this study who were not suitable for exercise and had medial history, such as congenital heart disease. Before the test, all the subjects should undergo a simple physical examination to ensure the safety of the subjects.

This study is divided into two parts. In the first stage, 200 subjects were tested for general physical indicators and power vehicle incremental load directly, and relevant indicators were collected for comparative correlation analysis, and then, data of 150 subjects were randomly selected. Try to add gender, age, height, weight, body mass index, quiet heart rate, and other independent variables to establish a regression equation to predict VO2max. In the second stage, the remaining 50 subjects were selected as the test group to test and evaluate the prediction effect of the prediction model.

#### 2.2.2. Main Indicators' Test Method

*(1) Heart Rate Measurement*. The heart rate of subjects was measured by RS800CXPolar and heart rate band was manufactured in Finland.

Test method is as follows. (1) Moisten the conductive pad with a little water, ensuring that the heart rate band is in close contact with the subject. (2) Then, find the position of the lower pectoral muscle of the participant and help him to wear the heart rate band to measure the heart rate. The looseness of the heart rate band can be adjusted freely. (3) After completing the above steps, adjust the polar table, and the value of the heart rate of the participants will appear in the table within two minutes. (4) When the heart rate of the participant appears in the table, the black heart rate chart will always shine, and the heart rate value will appear in time. (5) Participants were asked to sit quietly for five minutes while their heart rates were recorded.

*(2) Maximal Oxygen Uptake Test*. Adopt vertical power bicycle and METMAX3B portable gas analyzer for cardiopulmonary function test system.

Test steps are as follows. (1) Open the instrument and wait for half an hour of preheating, which is conducive to the test of the instrument. (2) Participants were fitted with a heart rate monitor and sat on a power bike in a quiet environment until the monitor remained stable. (3) Input the information required by the participants of the experiment and the experimental scheme. (4) Select the corresponding plan and then test the air around you. (5) Preparation of participants in the experiment: help them to wear breathing masks, install sensors, and then observe the changes in the heartbeat frequency and breathing data of participants in the experiment. After the preparation work is finished, the experiment can be carried out. (6) When the participants had no energy, the amount of oxygen absorbed was indicated. (7) Participants in the experiment complete the experiment.

### 2.3. Data Processing

All the measured data were processed by MicrosoftExcel2003 and SPSS20.0 statistical analysis software. All the data of the subject must be input into the form first. After the examination, all the data will be input into SPSS software, and all the data will be analyzed in this software. The test results of each index of the subjects were expressed as mean standard deviation ($\bar{x}\pm \text{SD}$). Finally, the correlation analysis between the predicted value of maximal oxygen uptake and the measured value of maximal oxygen uptake is carried out to test the correlation between them, so as to test the reliability of the calculation method. The significance level was defined as *P* < 0.05, and very significant level is defined as *P* < 0.01. In the multivariate linear regression analysis, firstly, the correlation between the measured indexes and VO2 max was analyzed, and the correlation and significance level between the indexes and VO2 max were analyzed. The gender, age, height, weight, BMI, resting heart rate, exhausted heart rate, maximum heart rate, and maximum load of the subjects were taken as independent variables, and gender was represented by virtual codes, making VO2 max a dependent variable for regression analysis, and the corresponding regression equation was obtained.

## 3. Result Analysis

### 3.1. Establishment of the Optimal Regression Equation for Predicting Maximal Oxygen Uptake

#### 3.1.1. Selection of Independent Variables

One hundred and fifty subjects of basic indicators and related indicators were in VO2 max test experiment with VO2 max correlation analysis; concrete analysis in Table 1 can be seen; to choose the high correlation with VO2 max and the correlation statistically significant indicators, then system analysis is carried out with these data, a clear correlation between their respective; this analysis is used as the basis for selecting the independent variables of the regression equation, see Table 1, and VO2 max index of significant correlation with sex, age, height, weight, BMI, maximum heart rate, and maximum load shows larger influence on the VO2 max index for gender, age, height, weight, BMI, maximum heart rate, and maximum load; these indicators are used in independent variable regression analysis.

#### 3.1.2. Establishment of the Optimal Regression Equation

VO2 max was selected as the dependent variable, and gender, age, height, weight, BMI, maximum heart rate, and maximum load were taken as independent variables for regression analysis. The five indexes of gender, weight, BMI, maximum heart rate, and maximum load in the data were entered into the regression equation, and the results of regression analysis are shown in Table 2 and Table 3.

As can be seen from Table 2, when VO2 max was the dependent variable and maximum load, body weight, gender, maximum heart rate, and BMI were the independent variables, the complex correlation coefficient (*R*) of model 5 was close to 0.9, indicating that the independent variables and dependent variables were closely related. The goodness of fit (*R*^2^) of simulation 5 is also close to 0.8, which fully proves that model 5 maintains a high degree of fit for samples, independent variables can explain the dependent variables well, and the model is meaningful for speculation [7]. It can be seen from Table 3 that the regression coefficients corresponding to the independent variables in the fifth row of the table are all less than 0.05, indicating that they are significant and can effectively predict the changes of dependent variables. Therefore, model 5 can be used as a method to calculate the maximal oxygen uptake of young people.

Max oxygen uptake = -0.784 + 0.009*∗* Max load +0.021*∗* Body weight +0.229*∗* Gender +0.004*∗* Max Heart rate +(-0.027) *∗*BMI (*R* = 0.884, *R*2 = 0.781, SEE = 0.205, and gender is represented by code: male = 0 and female = 1).

### 3.2. Back-Generation Test

All the data of 50 participants in the back-generation detection group were put into the equation to obtain the relevant predicted values, and then, the predicted and actual data were compared. The scatter diagram of the comparison results is shown in Figure 1, indicating that the predicted equation for calculating the maximum oxygen uptake of teenagers has a good linear relationship [8]. The results of further correlation analysis are shown in Table 4. It can be concluded that the correlation coefficient between the measured value of maximal oxygen uptake and the predicted value is 0.983, and the significance level is 0.000, which is significantly smaller than 0.01, indicating that there is an obvious concomitant relationship between the two. The high correlation between the predicted value and the measured value indicates that this formula can effectively predict the maximal oxygen uptake of teenagers.

### 3.3. Error Test

The error ratio between the measured maximal oxygen uptake value directly measured by power cycling test and the predicted value of 50 subjects in the test group was studied. The conclusion is shown in Figure 2. With the maximum load, maximum heart rate, body weight, and gender, BMI is taken as the independent variable, a regression model for the direct measurement of VO2 in 33 people's power cycle was established. The maximum percentage error between the measured values was less than 10%, 66% of the test sample to the generation of test sample size, within 15% of the 49 people, or 98% of the total test samples; only one person was above 15%, accounting for 2% of the total samples in the regression test.

## 4. Discussion

### 4.1. Index Selection for Establishing the Maximal Oxygen Uptake Equation

Physiologically speaking, VO2 max is related to cardiopulmonary function, muscle mass, activity status, and the ability to absorb and use oxygen. It is also influenced by genetic factors, age, gender, and exercise. During adolescence, the body develops rapidly, and some morphological indicators, such as height and weight, affect the development of maximal oxygen uptake to a certain extent. On the basis of these theories, this study selected gender, age, height, weight, BMI, resting heart rate, exhausted heart rate, maximum heart rate, and maximum load as independent variables that may be related to cardiopulmonary function [9]. It can be concluded from the results that VO2 max has the greatest correlation with maximum load, followed by weight, height, sex, BMI, and maximum heart rate. Finally, these indicators are selected as the independent variables of the regression equation.

### 4.2. Analysis of VO2 Max Inferred by the Regression Model

Through the above results obtained by stepwise regression analysis, we can get five regression equation models; in the five regression equation models, because the age range of subjects in this study is limited between 12 and 14 years old, there is no significant difference in age, height, fatigue, and heart rate among individuals. Therefore, the correlation between age and VO2 max in this study is not large. Height and exhaustion heart rate are still correlated with VO2 max to a certain extent, but there are multicollinearity problems between these two indicators and other indicators, which are eliminated in the process of stepped-regression analysis [10]. By comparing the correlation coefficients, the correlation coefficient between the regression equation and the maximal oxygen uptake was the highest in model 5, which was 0.884. By comparing their determination coefficients, the highest determination coefficient of model 5 is 0.781. By comparison of standard errors, the minimum standard error of model 5 is 0.205. By comparing the correlation coefficient, determination coefficient, and standard error between each model and VO2 max, it is recommended that the regression equation of VO2 max in this study is model 5 with maximum load, body weight, sex, maximum heart rate, and BMI as independent variables, which has the best measurement accuracy.

## 5. Conclusions

Taking maximum load, body weight, sex, maximum heart rate, and BMI as independent variables and maximum oxygen uptake as the dependent variable, the regression equation established in this study is as follows: maximum oxygen uptake = -0.784 + 0.009*∗* maximum load +0.021*∗* body weight +0.229*∗* sex +0.004*∗* maximum heart rate +(-0.027) *∗*BMI (*R* = 0.884, *R*2 = 0.781, SEE = 0.205, and gender is represented by code: male = 0 and female = 1). This study provides a new exploration direction for indirect estimation of maximal oxygen uptake. This new indirect test method has the advantages of high efficiency, low cost, fast, and convenient, requiring only simple measurement and moderate exercise intensity.

## Figures and Tables

**Figure 1:** Scatter diagram between the predicted maximal oxygen uptake and the measured maximal oxygen uptake (*n* = 50).

**Figure 2:** Error analysis of the predicted value and the measured value.

**Table 1:** Correlation coefficients between each index tested by the subjects and maximal oxygen uptake.

Indicators	Maximum oxygen uptake (L/min)

Gender	0.492^*∗∗*^
Age (years)	0.211^*∗∗*^
Height (cm)	0.591^*∗∗*^
Weight (kg)	0.662^*∗∗*^
BMI (kg/m^2^)	0.488^*∗∗*^
Quiet heart rate (sub/min)	0.013
The heart rate (sub/min)	0.198^*∗*^
Maximum heart rate (sub/min)	0.240^*∗∗*^
Peak load	0.754^*∗∗*^

^*∗∗*^, significant correlation at 0.01 level (bilateral); ^*∗*^, significant correlation at 0.05 level (bilateral).

**Table 2:** Regression model summary.

Model	*R*	*R* ^2^	Adjust *R*^2^	Standard error	Durbin–Watson

1	0.754a	0.568	0.565	0.285	
2	0.829b	0.687	0.683	0.243	
3	0.87c	0.756	0.751	0.215	
4	0.878d	0.771	0.765	0.209	
5	0.884c	0.781	0.774	0.205	1.604

**Table 3:** Coefficient.

Model		Nonstandardized coefficient		The standard coefficient	*t*	Sig
		B	Standard error	A trial version		

1	(Constant)	−0.131	0.14		−0.935	0.351
	The largest load	0.016	0.001	0.754	13.957	0
	(Constant)	0.399	0.125		−3.202	0.002
	The largest load	0.012	0.001	0.567	10.821	0

2	Weight	0.013	0.002	0.392	7.479	0
	(Constant)	−0.322	0.111		−2.993	0.003
	The largest load	0.011	0.001	0.526	11.222	0
	Weight	0.011	0.002	0.339	7.179	0

3	Gender	0.239	0.037	0.275	6.419	0
	(Constant)	−0.937	0.222		−4.212	0
	The largest load	0.01	0.001	0.48	9.993	0
	Weight	0.012	0.002	0.37	7.883	0
	Gender	0.237	0.036	0.272	6.531	0

4	Maximum heart rate	0.004	0.001	0.131	3.109	0.002
	(Constant)	−0.784	0.226		−3.467	0.001
	The largest load	0.009	0.001	0.435	8.665	0
	Weight	0.021	0.004	0.632	5.658	0

5	Gender	0.229	0.036	0.262	6.408	0
	Maximum heart rate	0.001	0.001	0.14	3.377	0.001
	BMI	−0.027	0.011	−0.261	−2.574	0.011

**Table 4:** Comparison of difference between measured and predicted values.

Maximum oxygen uptake measured value (L/min)	Estimated value of equation (L/min)	*r*

1.7722 ± 0.374	1.714 ± 0.393	0.983^*∗∗*^

^*∗∗*^, *P* < 0.01

## Data Availability

The data used to support the findings of this study are available from the corresponding author upon request.
